# Nursing Observation of Improved Administration Route of Protamine Sulfate Neutralizing Heparin

This article has been retracted.

**DOI:** 10.1155/2022/9334113

**Published:** 2022-03-08

**Authors:** Jia Hu, Suiting Zeng, Ziqi Wang, Qiuping Chen, Ya Shi, Yuanzhou Wu

**Affiliations:** ^1^Department of Ophthalmology, Zhujiang Hospital, Southern Medical University, Guangzhou 510280, China; ^2^Department of Anesthesiology Operation Room, Zhujiang Hospital, Southern Medical University, Guangzhou 510280, China; ^3^Department of Thoracic Surgery, Zhujiang Hospital, Southern Medical University, Guangzhou 510280, China

## Abstract

In this study, we have evaluated and examined various nursing effects of improved administration of protamine sulfate neutralizing heparin after cardiopulmonary bypass. For this purpose, retrospective analysis was made about the nursing records and clinical data of 216 patients who underwent cardiac operation under cardiopulmonary bypass in our hospital from January 2018 to December 2020. Among the enrolled patients, 118 patients were given subinterval administration of protamine sulfate neutralizing heparin via aortic root with the assistance of the scrub nurse at the end of cardiac surgery (improved group). A total of 98 patients were administered by the circulating nurse via the central vein (regular group). The changes of body temperature, blood pressure, oxygen saturation before and after heparin neutralization, and the total volume of thoracic drainage within 24 hours after operation were observed in the two groups, so as to evaluate the application effect of the improved administration of protamine sulfate neutralizing heparin from the perspective of nursing. There was no significant difference in age, gender, and other basic characteristics between the two groups (*P* > 0.05). The volume of drainage in the improved group and the regular group within 24 hours after surgery was 234 ± 26.3 ml and 307 ± 31.8 ml, respectively, *P* < 0.01, and the difference was statistically significant. The incidence of adverse reactions in the improved group was much lower than that in the regular group, *P* < 0.01. The administration route of the improved group was beneficial to maintain the stability of hemodynamics when using the protamine sulfate to neutralize heparin, which is worthy of clinical nursing promotion.

## 1. Introduction

Most cardiac operations require cardiopulmonary bypass (CPB). Heparin is still the preferred anticoagulant for cardiopulmonary bypass [1]. Protamine sulfate is a basic protein. It should be used after cardiac surgery to counteract the anticoagulant effects of heparin. In the process of neutralizing heparin, there are some adverse reactions related to protamine sulfate, but no reliable prevention methods have been found at present [2]. In our hospital, from January 2018 to December 2020, there were 216 patients who underwent cardiac operation under cardiopulmonary bypass (CPB). Surgical instrument nurses assisted the surgeon to administer protamine sulfate at intervals through the aortic root in 118 patients and 3 patients with protamine sulfate-related adverse events, the incidence rate was 2.5%, and the application effect was good. The results and the nursing experience report are as follows.

In this study, we have evaluated and examined various nursing effects of improved administration of protamine sulfate neutralizing heparin after cardiopulmonary bypass. For this purpose, retrospective analysis was made about the nursing records and clinical data of 216 patients who underwent cardiac operation under cardiopulmonary bypass in our hospital from January 2018 to December 2020. Among the enrolled patients, 118 patients were given subinterval administration of protamine sulfate neutralizing heparin via aortic root with the assistance of the scrub nurse at the end of cardiac surgery (improved group). A total of 98 patients were administered by the circulating nurse via the central vein (regular group). The changes of body temperature, blood pressure, oxygen saturation before and after heparin neutralization, and the total volume of thoracic drainage within 24 hours after operation were observed in the two groups, so as to evaluate the application effect of the improved administration of protamine sulfate neutralizing heparin from the perspective of nursing.

The remaining sections of this manuscript are arranged according to the following agenda items or paragraph which is given as follows.

In subsequent section entitled as Materials and Methods, the proposed mechanism is described in detail such as collection of data, nursing administration methods, observation, and statistical indexing methods. In Section 3, experimental results which are obtained after performing the experiment are presented along with detail discussion on how these results are obtained and how the proposed scheme is effective in resolving the aforementioned issues. A detailed discussion section is provided which described briefly how the proposed scheme is applicable in resolving the issue under consideration along with the relevant literature study. Finally, concluding remarks are provided at the end of the manuscript.

## 2. Materials and Methods

### 2.1. General Data

From January 2018 to December 2020, a total of 216 patients underwent cardiopulmonary bypass surgery. The clinical data of the patients were studied and analyzed. The patients were divided into two groups according to the different ways of nursing and administration of protamine sulfate neutralizing heparin. The scrub nurse assisted the surgeon to inject protamine sulfate through the aortic root intermittently (improved group). There were 118 patients in the improved group. There were 98 patients administered with protamine sulfate by the circulating nurse via the central vein (regular group).

### 2.2. Nursing Administration Method

Routine thoracotomy or thoracoscopic incision was performed, and heparin intravenous injection was done at a dose of 3 mg/kg bodyweight before the establishment of cardiopulmonary bypass. After the completion of heart surgery, the cardiopulmonary bypass was gradually stopped. After observing the stability of hemodynamic indexes, heparin was neutralized with protamine sulfate in a ratio of 1.2 : 1. In the improved group, protamine sulfate was administered at intervals. The surgical instrument nurse drew the medicine in the syringe and connected to the scalp needle. First, we slowly injected 20% protamine sulfate through the aortic root; then, we observed patient's blood pressure, heart rate, and blood oxygen saturation for 120 seconds. In the stable range, we continued to slowly inject the remaining 80% of protamine sulfate. In the routine group, protamine sulfate was injected slowly by the circulating nurse through the subclavian vein or internal jugular vein through the superior vena cava. Heparin (Chengdu Haitong Pharmaceutical Co., Ltd., batch no.: 191209) and protamine sulfate (Beijing Yuekang Pharmaceutical Group Co., Ltd., batch no.: 26080901Y) have the same source of supply and the same dosage ratio (protamine sulfate: heparin was 1.2 : 1).

### 2.3. Observation Indexes and Statistical Methods

The hemodynamic index of heparin neutralization was recorded during the whole administration of protamine sulfate. The patient's hemodynamic index included the changes of extremity temperature, blood pressure, oxygen saturation, and total amount of drainage fluid within 24 hours after operation and so on. The paired *t*-test was used for measurement data, and the chi-square test was used for enumeration data. *P* < 0.05 was considered as statistically significant.

## 3. Experimental Results and Observations

### 3.1. Basic Characteristics of Patients

The ages of the modified group and the conventional group were 17–76 years old (median age 58 years old) and 21–79 years old (medium age 59 years old), respectively. There were 48 males (27 in the improved group and 21 in the conventional group) and 57 females (31 in the improved group and 26 cases in the conventional group). The body mass index (BMI) of the patients in the two groups was 22 ± 3 and 22 ± 4, respectively. There was no statistical difference in the above indicators between the two groups, as given in Table 1.

### 3.2. Adverse Reactions of Protamine Sulfate in Two Administration Routes

In the administration process of protamine sulfate, nurses should closely observe the patient's limb temperature, blood pressure, and saturation of pulse oxygen. Drug-induced reactions can be divided into mild and severe levels according to the changes of the above indicators [3, 4]. In this study, more patients in the improved group had no clinical features (67/118 vs. 35/98) in the improved group, and the difference was statistically significant, *P* < 0.01. There were 48 cases of mild reaction and 54 cases of mild reaction, respectively, and there was no statistical difference between the two groups (*P* > 0.05). Among the patients with severe protamine adverse reactions, 3 cases were in the modified group. They had significant decrease in blood pressure and slow heart rates. In the conventional group, there were 9 patients with severe protamine adverse reactions, including 5 cases with decreased blood pressure, 2 cases with bradycardia, and 2 cases with airway resistance increased, and the difference was statistically significant, *P* < 0.05, as given in Table 2.

### 3.3. Modified Group

In this group, we slowly injected 20% protamine sulfate through the aortic root first; then, we observed patient's blood pressure, heart rate, and blood oxygen saturation for 120 seconds and continued to slowly inject the remaining 80% of protamine sulfate. In the routine group, protamine sulfate was injected slowly by the circulating nurse through the subclavian vein or internal jugular vein through the superior vena cava. The ACT values of patients in the two groups were recorded 10 minutes before operation (basic ACT), 5 minutes after heparinization, and 5 minutes, 30 minutes, 60 minutes, and 180 minutes after neutralization, and the results are given in Table 3.

### 3.4. Recording of Data

We recorded the length of operation time and the median drainage volume within 24 hours. The retention time of drainage tube and thoracotomy for hemostasis were also recorded. In the improved group, the median 24 hour drainage volume after the neutralization of heparin with protamine sulfate was 261 ml, significantly less than the conventional group (307 ml, *P* < 0.01), as given in Table 4. All of these resulted in the better outcomes in the improved group, including the less duration of use of pressor (*P* < 0.01), the higher LVEF 24 hours after surgery (*P* < 0.05), as given in Table 5.

## 4. Nursing Experience and Discussion

Protamine sulfate is a cationic low molecular protein compound extracted from fresh and mature fish sperm, which inactivates heparin by combining with heparin to form a neutral complex after injection into blood circulation, so it has been widely used in heart and vascular surgery to reverse the anticoagulant effect of heparin [5, 6].

The adverse reactions of protamine sulfate have long been confirmed. If the intravenous injection rate is too fast, it can cause hypotension, bradycardia, pulmonary hypertension, dyspnea, and other adverse reactions, with the reported incidence ranging from 0.06% to 10.6% [7]. Most heart disease patients are heavier and older, and some patients are complicated by a variety of basic diseases, poor preoperative general situation, patients with anesthesia and surgery tolerance level is poorer, so nursing is given before and after surgery in supervision to fully understand the patients with or without food or drug allergy history, especially pay attention to the presence of preoperative renal failure in patients needing blood dialysis [8]. According to statistics, the incidence of cataclysmic adverse reaction events related to protamine sulfate ranges from 0.28% to 2.6%, and once the occurrence occurs, the patients will face a great risk with a total mortality rate of 2–2.6% [9].

For critically ill patients with cardiovascular disease in extracorporeal circulation cardiac surgery, the intraoperative extracorporeal circulation group of physicians and anesthesiologists using drugs is various, nursing staff should carefully check the name of the drug to verify the specification of protamine and records of heparin and protamine sulfate manufacturer and serial number, according to patients' weight to accurately calculate the dose good to use. Before neutralizing heparin with protamine sulfate, routine intravenous administration of dexamethasone and calcium gluconate was used to prevent allergic reactions. The method of intermittent administration of protamine sulfate through the aortic root and slow injection of 20% dose in the first 5 min is beneficial to observe whether there is drug-induced hypersensitivity reaction. After the elimination of adverse reactions, the administration continues. Protamine directly binds to heparin in the systemic circulation, which can reduce the amount of protamine entering the pulmonary circulation. It can reduce the release of inflammatory mediators such as histamine and 5-hydroxytryptamine in lung tissue and reduce the occurrence of adverse reactions to a certain extent [10].

In our study, the incidence of severe adverse reactions in the modified protamine sulfate administration pathway group was reduced to 3.4%, while that in the conventional group was 17%, suggesting that improved nursing measures including optimizing the protamine administration pathway can reduce the occurrence of adverse reactions in the protamine sulfate group (*P* < 0.05). At the same time, we found that the median amount of drainage fluid 24 hours after surgery in the conventional group was 307 ml, which was significantly higher than that in the improved group (*P* < 0.001), and the possible reason was analyzed to be related to the drug treatment after the increase of pulmonary artery pressure caused by protamine.

## 5. Conclusion

In this study, we have evaluated and examined various nursing effects of improved administration of protamine sulfate neutralizing heparin after cardiopulmonary bypass. For this purpose, retrospective analysis was made about the nursing records and clinical data of 216 patients who underwent cardiac operation under cardiopulmonary bypass in our hospital from January 2018 to December 2020. Among the enrolled patients, 118 patients were given subinterval administration of protamine sulfate neutralizing heparin via aortic root with the assistance of the scrub nurse at the end of cardiac surgery (improved group). A total of 98 patients were administered by the circulating nurse via the central vein (regular group). The changes of body temperature, blood pressure, oxygen saturation before and after heparin neutralization, and the total volume of thoracic drainage within 24 hours after operation were observed in the two groups, so as to evaluate the application effect of the improved administration of protamine sulfate neutralizing heparin from the perspective of nursing. Finally, this study found that the modified administration of intermittent administration of protamine sulfate and heparin via the aortic route resulted in a lower incidence of protamine-related adverse reactions and less postoperative drainage volume in patients, which was a safer administration method for protamine sulfate and heparin.

## Figures and Tables

**Table 1:** General information of the two groups of patients with different administration routes of protamine sulfate.

Basic characteristics	Improved group (*N* = 118)	Regular group (*N* = 98)	*P* value
Age (y)			
Median (mix, max)	58 (17.76)	59 (21. 79)	>0.05
Gender			
Male	57	42	>0.05
Female	61	56	
BMI (kg/m^2^)	22 ± 3	22 ± 4	>0.05
Cardiac function grading^*∗*^ (NYHA)			
I	2	1	>0.05
II	22	23	
III	61	56	
IV	33	18	

^*∗*^Cardiac function grading: the stages of heart failure are according to The New York Heart Association (NYHA) classification.

**Table 2:** Comparison of the incidence of drug-induced reactions between the two protamine sulfate administration routes.

Drug-induced reactions	None	Mild	Severe
Improved group (*N* = 118)	67	48	3
Regular group (*N* = 98)	35	54	9
*P* value	<0.01	>0.05	<0.05

**Table 3:** Comparison of ACT results between two groups at each point in time.

ACT results (min)	Improved group	Regular group	*P* value
−10 (*s*)^a^	116.63 ± 10.23	117.52 ± 11.17	>0.05
5 (*s*)^b^	556.86 ± 25.23	562.32 ± 30.64	>0.05
5 (*s*)^c^	112.63 ± 18.26	123.23 ± 20.26	>0.05
20 (*s*)^c^	115.66 ± 17.63	131.23 ± 18.36	<0.05
30 (*s*)^c^	110.23 ± 14.82a	122.23 ± 20.47	<0.05
60 (*s*)^c^	115.32 ± 18.16	116.30 ± 18.51	>0.05
180 (*s*)^c^	113.63 ± 18.23	116.33 ± 20.03	>0.05

^a^The ACT value 10 minutes before operation (basic ACT value). ^b^The ACT value 5 minutes after heparinization. ^c^The ACT value 5 minutes, 30 minutes, 60 minutes, and 180 minutes after neutralization, respectively.

**Table 4:** The influence of two administration routes on blood coagulation function.

Administration routes	Improved group	Regular group	*P* value
The length of operation time (h)	191.06 ± 5.23	189.06 ± 8.82	>0.05
Median drainage volume within 24 hours (ml)	261 ± 26.3	307 ± 31.8	<0.01
Retention time of drainage tube (h)	38.78 ± 6.02	41.74 ± 6.52	>0.05
Thoracotomy for hemostasis (*n* (%))	0 (0)	1 (1)	>0.05

**Table 5:** Comparison of safety indicators between two administration routes after data matching.

Administration routes	Improved group	Regular group	*P* value
Duration of use of pressors (h)	30.38 ± 1.26	36.06 ± 2.22	<0.01
Length of stay in ICU (d)	1.88 ± 0.16	2.02 ± 0.18	>0.05
LVEF 24 hours after surgery (%)	51.88 ± 3.16	48.02 ± 4.18	<0.05
Total length of stay (d)	15.92 ± 6.12	15.88 ± 7.46	>0.05

## Data Availability

The datasets used and analyzed during the current study are available from the corresponding author upon request.
